# Mechanism of Action of the Novel Nickel(II) Complex in Simultaneous Reactivation of the Apoptotic Signaling Networks Against Human Colon Cancer Cells

This article has been retracted.

**DOI:** 10.3389/fphar.2015.00313

**Published:** 2016-01-28

**Authors:** Nima Samie, Batoul Sadat Haerian, Sekaran Muniandy, Anita Marlina, M. S. Kanthimathi, Norbani B. Abdullah, Gholamreza Ahmadian, Raja E. R. Aziddin

**Affiliations:** ^1^Department of Pharmacology, Faculty of Medicine, University of MalayaKuala Lumpur, Malaysia; ^2^Drug and Research Unit, Department of Pathology, Hospital Kuala LumpurKuala Lumpur, Malaysia; ^3^Department of Molecular Medicine, Faculty of Medicine, University of MalayaKuala Lumpur, Malaysia; ^4^Department of Chemistry, Faculty of Science, University of MalayaKuala Lumpur, Malaysia; ^5^Faculty of Medicine, University of Malaya Centre for Proteomics Research, University of MalayaKuala Lumpur, Malaysia; ^6^Department of Environmental and Industrial Biotechnology, National Institute of Genetic Engineering and BiotechnologyTehran, Iran

**Keywords:** apoptosis, cell cycle arrest, nickel(II) complex, NF-κB, colon cancer

## Abstract

The aim of this study was to evaluate the cytotoxic potential of a novel nickel(II) complex (NTC) against WiDr and HT-29 human colon cancer cells by determining the IC_50_ using the standard MTT assay. The NTC displayed a strong suppressive effect on colon cancer cells with an IC_50_ value of 6.07 ± 0.22 μM and 6.26 ± 0.13 μM against WiDr and HT-29 respectively, after 24 h of treatment. Substantial reduction in the mitochondrial membrane potential and increase in the release of cytochrome c from the mitochondria directed the induction of the intrinsic apoptosis pathway by the NTC. Activation of this pathway was further evidenced by significant activation of caspase 3/7 and 9. The NTC was also shown to activate the extrinsic pathway of apoptosis via activation of caspase-8 which is linked to the suppression of NF-κB translocation to the nucleus. Cell cycle arrest in the G1 phase was confirmed by flow cytometry and up-regulation of glutathione reductase expression was quantified by qPCR. Results of the current work indicates that NTC possess a potent cancer cell abolishing activity by simultaneous induction of intrinsic and extrinsic pathways of apoptosis in colon cancer cell lines.

## Introduction

Colon cancer is the third common type of cancer and the second foremost cause of cancer death when both sexes are pooled (Siegel et al., 2015). Following failure of normal replacement of lining cells in the colon, cells begin to divide abnormally which results in formation of polyps. As polyps grow, further genetic mutations destabilize the cells to invade other layers of the colon. Despite significant diagnostic strategies in colon cancer and application of different modalities, including surgery, chemotherapy, and radiotherapy, the relapse and metastasis are still considered incurable and the 5-year relative survival rate is approximately 15% (Ferlay et al., 2014).

Apoptosis has been predominantly considered as one of the most important targets in anti-cancer therapy. This signaling pathway has a fundamental role in the emergence of cancer and the patient's response to treatment (Lowe and Lin, 2000). Apoptosis promotes the process of programmed cell death through the extrinsic and/or mitochondrial (intrinsic) pathways, regulated by a number of gene families. By contrast, activation of the extrinsic pathway is through the cell surface death receptors, whereas the intrinsic pathway can be independently induced by an extensive array of signals such as cytotoxic drugs, cellular stress, and radiation. Defect in these pathways can endorse neoplastic development or resistance to anticancer therapies (Kranz and Dobbelstein, 2012). Targeting the key proteins involved in apoptosis signal transduction can improve cell death and thus overcome the clinical consequence in cancer therapy. They are including PI-3K/Akt (Huang et al., 2001), HIF-1α (Viemann et al., 2007), NF-κB (Chen et al., 2001; Huang et al., 2002; Cruz et al., 2004), AP-1 (Wisdom, 1999; Cruz et al., 2004), and NFAT(Huang et al., 2001; Cai et al., 2011) by influencing the expression pattern of transcription factors and inducing epigenetic mechanisms such as DNA methylation, loss of histone acetylation rather than indirect DNA damage (Salnikow and Zhitkovich, 2007; Arita and Costa, 2009).

The water-soluble nickel salts are less toxic than water-insoluble compounds (Cempel and Nikel, 2006). The potency of nickel compounds is related to the ability of Ni^2+^ to access chromatin, where it produces an increased chromatin condensation, enhanced DNA methylation, and turning off of the transcription of tumor suppressor and senescence genes (Zhou et al., 1998). Following the entry into the cell, nickel compounds stimulate generation of reactive oxygen species (ROS) which cause multiple types of cellular and nuclear damage either through direct or indirect mechanisms (Salnikow et al., 2000; Waris and Ahsan, 2006). The aim of this study is to evaluate the cytotoxic properties of a novel nickel(II) complex (NTC) against human colon cancer cells through targeting apoptotic pathways.

## Materials and methods

### Reagents and chemicals

All chemicals are commercially available and used as received. The elemental analyses for C, H, and N were carried out on a Thermo Finnigan Flash EA 1112 (Thermo Scientific, Hudson, NH, USA). The infrared spectra were obtained on a Perkin-Elmer Spectrum 400 spectrometer with samples as KBr pellets in the region 4000–400 cm-1. The UV-vis spectra were obtained using a Shimadzu UV-vis-NIR 1600 spectrophotometer. ^1^H-NMR spectra were recorded on a JEOL FT-NMR lambda 400 MHz spectrometer. The solvent was DMSO-d_6_. The chemical shifts were reported in ppm using the residual protonated solvent as the reference.

### General procedure of synthesis of the thiophene-based ligand (L)

2, 4-Diamino-6-phenyl-1, 3, 5-triazine (18.89 g; 100.9 mmol) was added portionwise to a solution of 2, 5-thiophenedicarboxylic acid (12.93 g; 100.9 mmol) in absolute ethanol (100 mL). The mixture was refluxed for 2 h and then left to cool to room temperature. The white powder formed was filtered, washed with ethanol and dried in an oven at 80°C. The yield was as follows 31.15 g, 97.9%. ^1^H NMR (400 MHz, DMSO-*d*_6_): δ = 8.23–8.25 (d, 2H, ar-H3), 7.71 (s, 1H, NH), 7.44–7.51 (m, 2H, ar-H1, H-2), 6.80 (b, 2H, ar-H4). Anal.calc. for C_15_H_11_N_5_O_3_S: C, 52.8; H, 3.3; N, 20.5. Found: C, 52.6; H, 3.9; N, 20.7. Formula weight, 341.34 g mol^−1^. IR, cm^−1^: 3324 (N-H), 1672 (C=O amide).

### Synthesis of Ni (II)-complex with thiophene based ligand

Nickel(II) hexadecanoate (0.80 g; 1.4 mmol) was added to an ethanolic suspension of L (0.48 g; 1.4 mmol), and the mixture was heated under reflux for 3 h. The greenish powder formed was filtered from the hot reaction mixture, washed with ethanol, and dried in an oven at 100°C. Yield: (0.84 g, 65.6%). Anal. calc. for Ni_2_C_79_H_133_N_5_O_10_S: C, 64.9; H, 9.2; N, 4.8. Found: C, 64.6; H, 9.4; N, 4.1. Formula weight, 1462.38 g mol^−1^. IR, cm^−1^: 3326 (N-H), 2916 (CH_2asy_), 2849 (CH_2sym_), 1617 (C=O amide), 1525 (COO_asy_), 1395 (COO_sym_), 569 (Ni-N).

### Cell lines and cell culture

The human colon cell line, CCD-18Co, and colon cancer cell lines, WiDr and HT-29, were purchased from the American Type Culture Collection (ATCC, Manassas, Virginia, USA). WiDr and CCD-18Co cells lines were cultured in Eagle's Minimum Essential Medium and HT-29, in RPMI-1640 supplemented with 10% heat inactivated fetal bovine serum (FBS, Sigma-Aldrich, St. Louis, MO), 1% penicillin and streptomycin. All cell lines were cultured in a humidified incubator with 5% CO_2_ at 37°C. All experiments were conducted on cell lines with passage number 1–10.

### Cell proliferation assay

The MTT [3-(4, 5-dimethylthiazol-2-yl)-2, 5-diphenyltetrazolium bromide] assay was carried out to evaluate the anti-proliferative activity of the nickel(II) complex (NTC). Briefly, cells were seeded (100 μl) 24 h prior to treatment in a 96-well plate at 7 × 10^4^ cells/ml. NTC and 5-fluoruracil as control positive were dissolved in 0.1% DMSO (Sigma Chemical Co., St. Louis, Missouri, USA). After incubation of the plates for 24, 48, and 72 h at 37°C with 5% CO_2_, 50 μl of MTT solution (2 mg/ml; Sigma) was added to each well and then plates were incubated for 4 h at the same conditions. To dissolve the purple formazan crystals formed at the bottom of the wells, 100 μl DMSO was added to each well and incubated for 20 min. Absorbance was subsequently read at 570 nm using a spectrophotometric plate reader (Hidex, Turku, Finland). The dose-response curves were plotted to obtain the IC_50_ values. Experimental data were derived from three independent experiments. The selectivity index was obtained by mean IC_50_ CCD-18Co/mean IC50 of WiDr or HT-29.

### Measurement of the released LDH

Quantitative measurement of lactate dehydrogenase (LDH) released into the media from damaged cells as a biomarker for cellular cytotoxicity and cytolysis was carried out according to Wang et al. (2014) with slight amendment. Briefly, cells were treated with different concentrations of NTC and Triton X- 100 (positive control) for 48 h followed by transfer of the supernatants of untreated and treated cells to a new 96-well plate for LDH activity analysis. 100 μL of LDH reaction solution was then added to each well, followed by incubation at room temperature for 30 min. The absorbance was read at 490 nm using a Tecan Infinite 200 Pro (Tecan, Mannedorf, Switzerland) microplate reader. LDH activity of the cells was assessed by the amount of formazan salt and intensity of red color in treated and untreated samples. Release of LDH level in treated cells was expressed as a percentage of LDL release in the positive control.

### Immunofluorescence

After 24 h NTC treatment of both cancer and normal cells, mitochondrial membrane potential (MMP) and cytochrome c release were analyzed using JC-1 assay kit (Life Technologies, Gaithersburg, MD, USA) and ApoTrack cytochrome c apoptosis ICC antibody kit (Abcam Inc., Cambridge, MA, USA), respectively, according to the manufacturer's protocol. Cells were then fixed in 4% paraformaldehyde, permeabilized by 0.25% Triton X-100 and then were quenched with 50 mM ammonium chloride and blocked with 5% BSA in PBS overnight, followed by probing with 10 μg/mL DY350-Phalloidin and 4 μg/mL Hoechst 33,342 (Thermo Scientific, Hudson, NH, USA) and was incubated at room temperature for 20 min. Finally, cells were washed with PBS and coverslips were mounted using polyvinyl alcohol mounting medium (Fluka Analytical, Milan, Italy). Fluorescence was analyzed using the Radiance 2100 confocal microscope (Bio-Rad, Hercules, CA, USA). Noise reduction was attained by Kalman filtering during application and data was analyzed with Data Viewer version 3.0.

### Annexin-V-FITC assay

Cells were treated with cell membrane permeable calcium chelator (EGTA/AM, 25 mM, Life Technologies, Gaithersburg, MD, USA) for a period of 1 h prior to addition of NTC (6.0 μM). After 24 h treatment, cells were harvested, washed twice with PBS, resuspended in Annexin-V binding buffer (BD Biosciences, San Jose, CA, USA) and stained with Annexin-V-FITC (BD) and PI (Sigma) according to the manufacturer's protocol. The fluorescence intensity was then examined using FACSCanto II (BD Biosciences, San Jose, CA). Onset of early and late apoptosis were determined using Annexin-V, whereas PI was utilized for distinguishing necrosis and late apoptosis.

### Determination of apoptotic properties

Accurate determination of live/dead nucleated cell concentration in the sample was accomplished by the minor modified version of the method described by Rahman et al. (2014). Propidium iodide (PI) and acridine orange (AO) double staining assay was performed to detect the early and late apoptotic properties of the treated cancer cells according to the standard procedure. Cells were incubated with NTC (6.0 μM) for 24, 48, 72 h and the harvested cells were stained with acridine orange and propidium iodine and observed within 30 min with a UV-fluorescent microscope (Bio-Rad, Hercules, CA, USA).

### ORAC antioxidant assay

Organisms have complex antioxidant systems to protect themselves from oxidative stress; however, excess oxidative stress can overwhelm the systems and cause severe damage. To measure the antioxidant protection potential of NTC over time, the ORAC assay was used. In a black 96-well plate, 6.0 μM of NTC, blank (solvent/PBS) and standard (5-fluouracil) were added to cells supplemented with fluorescein solution (150 μL) and incubated at 37°C for 5 min. AAPH (25 μL) was then added and fluorescence intensity was assessed at 485 nm (excitation wavelength) and 538 nm (emission wavelength) every 2 min for a duration of 2 h. Quantification was carried out by calculating the differences of area under the fluorescence decay curve of the samples and blank.

### Detection of ROS production

ROS is produced as byproducts during the mitochondrial electron transport and has potential to cause apoptosis. Production of intracellular ROS was detected by using 10 mM dihydroethidium (DHE) stock solution (in methanol) diluted 500-fold in HBSS without serum or other additives to yield a 20 mM working solution. The cells in the black plate were washed twice with HBSS after exposure to NTC and then incubated in 100 μL working solution of DHE at 37°C for 30 min. Fluorescence of DCF in each cell was captured, extracted and analyzed with Radiance 2100 confocal microscope (Bio-Rad, Hercules, CA, USA).

### Evaluation of NF-κB translocation

Nuclear factor kappa-light-chain-enhancer of activated B cells controls transcription of DNA and is involved in cellular responses to stimuli such as stress, free radicals and chemicals. Cells were treated with NTC (6.0 μM) and stimulated with TNF-α. The cells were then stained according to the instructions of the Cellomics nuclear factor-kB (NF-κB) activation kit (Thermo Scientific). The cytoplasmic and nuclear NF-κB intensity ratio (average intensity of 200 cells/well) was measured using cytoplasm to nucleus translocation bio-application software (S50-5001-1, Thermo Scientific).

### Gene expression analysis

WiDr and HT-29 cells were treated with NTC (6.0 μM) for 24 h. Total RNA was extracted using RNeasy plus mini kit (Qiagen). Reverse transcription of 1 mg RNA into cDNA was carried out by using RT2 first strand kit (SA Biosciences, Qiagen). RT2 Real Time TM SYBR Green/fluorescein PCR master-mix was then mixed with cDNA and loaded into each of 96 wells of the 84 genes by qPCR array according to the manufacturer's protocol (SA Biosciences, Qiagen). Differential expression of the members of antioxidant peroxiredoxin (PRDX) family and redox control are involved in human oxidative stress and cellular stress response were analyzed. Concisely, 12.5 ml master mix, 11.5 ml double distilled water, and 1 ml cDNA was mixed to reach the final volume of 25 ml PCR mixture and 25 μl was loaded to each individual well of the 96 well plate. QuantStudio™ 12K Flex Real-Time PCR System (Life Technologies, Bleiswijk, Netherlands) consuming ssoFast EvaGreen Supermix (Bio-Rad) was operated according to the manufacturer's protocols. Primers were synthesized as GR F5′-AACATCCCAACTGTGGTCTTCAGC-3′, GR R5′-TTGGTAACTGCGTGATACATCGGG-3′, β-actin F5′-GATGACCCAGATCATGTTTGAGACC-3′ and β-actin R5′-AGTCCATCACGATGCCAGTGGT-3′. Amplification was operated at 95°C for 10 min, followed by 40 cycles at 95°C for 15 s and 60°C for 1 min. The average expression of five housekeeping genes including β-actin (ACTB), β-2-microglobulin (B2M), hypoxanthine phosphoribosyltransferase 1 (HPRT1), ribosomal protein L13a (RPL13A) and glyceraldehyde-3-phosphate dehydrogenase (GAPDH) was considered for normalization of mRNA expression of each gene. Difference in gene expression between piperazine and untreated control was calculated by the RT Profiler qPCR-array data analysis software to measure the fold changes.

### Evaluation of mitochondrial and extrinsic apoptotic pathways

Caspases are a family of cysteine proteases that have critical roles in apoptosis. Caspase 8 is involved in mitochondrial (intrinsic) whereas, caspase 8 in the extrinsic pathway of apoptosis. Caspase 3 interacts with caspase-8 and caspase-9 and plays a central role in the execution-phase of cell apoptosis. Time-dependent evaluation of caspase-3/7, -8, and -9 activities in the presence of NTC (6.0 μM) were performed using assay kits Caspase-Glo 3/7, 8, and 9 (Promega Corp., Madison, WI, USA) in triplicates on white 96-well after 6, 12, 18, 24, and 30 h. Treatment of the cells with NTC (6.0 μM) was carried out 24 h prior to the experiment on a total of 10,000 cells per well. A 100 ml of the caspase-Glo reagent added and incubated at room temperature for 30 min. The substrate of luciferase enzyme will be released from apoptotic cells due to caspase activation after cleavage of the aminoluciferin-labeled synthetic tetrapeptide. Caspase activities were measured using Tecan Infinite 200 Pro (Tecan, Mannedorf, Switzerland) microplate reader.

### Molecular identification of apoptotic proteins induced by NTC

Apoptotic proteins have central role in regulation of programmed cell death via inducing (pro-apoptotic) or inhibiting (anti-apoptotic) apoptosis. 1 × 10^6^ cells/mL were treated with NTC and standard (5-fluorouracil) separately for 24 h. One milliliter of cells were then aspirated, lysed in 300 μl of Tris-HCL buffer and resolved on 10% SDS-polyacrylamide gels followed by transferring of the proteins to PVDF membranes (Millipore) and blocking with 5% non-fat dry milk in PBS- T (0.05% Tween 20) for 1 h at room temperature. Primary antibodies including Bid (sc-11243, 1:1000), caspase-3 (sc-7148, 1:1000), caspase-8 (sc-56070, 1:1000), caspase-9 (sc-56076, 1:1000), anti β-actin (sc-47778, 1:5000), Bax (sc-23959, 1:1000) Santa Cruz Biotechnology Inc. (Santa Cruz, CA, USA), Bcl-X_L_ (ab32370, 1:1000), Bcl-2 (ab7973, 1:1000), and p53 (ab2433, 1:1000) (Abcam Inc., Cambridge, MA, USA). Secondary antibodies conjugated to horseradish peroxidase were obtained from Kirkegaard & Perry Laboratories, Inc. (Gaithersburg, MD, USA). Protein-antibody complexes were detected using Amersham ECL prime Western blotting detection reagent (GE Healthcare, Munich, Germany).

### Statistical analysis

All values are expressed as mean ± S.D. Student's *t*-test was used for statistical evaluation of data. Probability values ^*^p < 0.05 were considered statistically significant.

## Results

### Structure elucidation

The synthetic steps for the preparation of ligand (*L*) is shown in Figure 1A. The structural formula of *L* was ascertained from ^1^H-NMR and FTIR spectroscopies. The ^1^H-NMR spectrum supported the proposed structural formula (Figure 1B). The amide protons appear as a singlet at 7.71 ppm, and all aromatic protons appear as a multiplet in the range 7.44–7.51 ppm. Ni (II) complex containing polymeric ligand was synthesized as a greenish precipitate in ethanolic solution owing to their low ethanol solubility (Figure 1C). The complex is a dinuclear repeat unit and stable toward air and moisture. It is soluble in DMSO but insoluble in common organic solvents. The FTIR spectra of *L* and its complex showed a broad band at 3324 cm^−1^ and 3326 cm^−1^ that is assigned ν (N-H) amide. FTIR spectra of *L* showed the absence of bands of ν(C=O) and ν(NH_2_), which were present in the starting material. It is due to the formation of an amide bond ν(C=O) that indicates the condensation of the two moieties (a carboxylic acid monomer and an amine monomer). Its complex showed a weak band at low frequency 569 cm^−1^, revealing the coordination between nickel ion and nitrogen atom of the ligand. The ΔCOO value (COO_asy_–COO_sym_) of its complex was 130 cm^−1^, suggesting a chelating binding mode for carboxylate coordination mode. The UV-visible spectrum of Ni (II) complex indicates the octahedral geometry at Ni (II) center.

**Figure 1:** **(A)** The synthetic steps for the preparation of ligand. **(B)** The structural formula of *L* was ascertained from ^1^H-NMR and FTIR spectroscopies. The amide protons appear as a singlet at 7.71 ppm, and all aromatic protons appear as a multiplet in the range 7.44–7.51 ppm. **(C)** Ni (II) complex containing polymeric ligand was synthesized as a greenish precipitate in ethanolic solution owing to their low ethanol solubility. The complex is a dinuclear repeat unit and stable toward air and moisture. It is soluble in DMSO but insoluble in common organic solvents.

### Cytotoxic effect of NTC on proliferation of cancer cells

The cytotoxic effect of NTC was evaluated on WiDr and HT-29 and CCD-18Co by the MTT assay in triplicate. IC_50_ values for the compound and standard on cell lines tested in this work are shown in Table 1. The NTC displayed a very significant inhibitory effect toward both cancer cells after 24 h. The IC_50_ of NTC against WiDr and HT-29 were calculated as 6.07 ± 0.22 μM and 6.26 ± 0.13 μM, respectively, as compared with the standard (1.04 ± 0.14) but the IC_50_ of NTCin normal cells was 55.16 ± 0.07 μM.

**Table 1:** **MTT cell proliferation assay for 24, 48, and 72 h on normal and cancer cells**.

**Time (h)**	**WiDr**	**HT-29**	**CCD-18Co**
**IC_50_ (μM) of nickel(II) complex (NTC)**			
24	6.07 ± 0.22	6.26 ± 0.13	55.16 ± 0.07
48	5.87 ± 0.35	6.02 ± 0.02	53.25 ± 0.11
72	5.65 ± 0.11	5.91 ± 0.23	52.94 ± 0.06
**IC_50_ (μM) of 5-fluoruracil (5-FU)**			
24	1.08 ± 0.14	1.17 ± 0.06	1.33 ± 0.15

### NTC induced G1 cell cycle arrest

Development of cancer is due to dysfunction in the regulation of the cell cycle that results in over-proliferation of cells. However, cancer progression can be strongly limited by conquest of the cell cycle. Hence, the effect of 6.0 μM NTC on cell cycle arrest was investigated. The BrdU and phospho-histone H3 staining of HT-29 and WiDr cells treated with NTC showed that cell cycle arrest at the S/M phases did not occur (Figure 2). However, cellular arrest in the G1 phase was detected by using flow cytometry (Figure 3).

**Figure 2:** **NTC arrests the cell cycle in the S/M phase**. Cells were incubated with DMSO (control negative) and NTC (6.0 μM) for 24 h following collection and staining with BrdU and Phopho-Histone H3. Treatment with NTC revealed no significant changes in the BrdU and Phosho-Histone H3 fluorescence intensity which suggests that the cells have not been arrested at S/M phase.

**Figure 3:** **Effect of NTC on development of cell cycle using flow cytometry**. Momentous cell cycle arrest was identified at G1 phase after 24 and 48 h incubation of the cells with NTC. All data were expressed as the means ± standard error of triplicate measurements. ^*^P < 0.05 compared with the no-treatment group.

### NTC enhanced cytochrome C release and membrane permeability but reduced mitochondrial membrane potential

Because of the cytotoxic effect of NTC on WiDr and HT-29 cells, the membrane permeability was much higher than the control suggesting sustained apoptotic activity in these cells (Figure 4A). Loss of mitochondrial membrane potential (MMP) is a conceivable mechanism for cell death evidenced by MMP dye (JC-1) which stained control cell cytoplasm stronger than cells treated with NTC. The WiDr and HT-29 cells treated with NTC for 24 h exhibited a dose-dependent reduction of MMP fluorescence intensity, as a result of collapsed MMP. The fluorescence intensity in the cytosol of WiDr and HT-29 cells treated with NTC was less than control cells suggesting the release of cytochrome c. In addition, increase in the plasma membrane permeability was evidenced by increase in the green fluorescent intensity of NTC-treated cancer cell lines (Liew et al., 2014) which confirm that NTC disturb the plasma membrane and increase the permeability as result of its cytotoxic potential (Figures 4A,B).

**Figure 4:** **Immunofluorescence study of the effect of NTC. (A)** After treatment of the cells with NTC (6.0 μM), Hoechst 33,342, cytochrome c, membrane permeability and mitochondrial membrane potential dyes were applied. **(B)** Representative bar charts indicate a dose-dependent reduction of MMP (JC-1), elevated cell permeability and cytochrome c release in treated cells. All data were expressed as the means ± standard error of triplicate measurements. ^*^P < 0.05 compared with the no-treatment group.

### Cytoskeletal rearrangement and nuclear fragmentation

WiDr and HT-29 cells treated with NTC were examined for cytoskeletal and nuclear morphological alteration by phalloidin and Hoechst 33,342 staining. Staining of F-actin at the peripheral membrane showed cell shrinkage (Supplementary Figure 1). Nuclear condensation and fragmentation were detected at a concentration of 6.0 μM of NTC in 24 h (Supplementary Figure 2). Additionally, apoptotic chromatin changes increased nuclear intensity which suggested that NTC induced apoptosis in these cells (Liew et al., 2014).

### Morphological changes in the NTC-induced apoptosis cells

After 24 h treatment of WiDr and HT-29 cells with 6.0 μM of NTC, the apoptotic features were analyzed by using a fluorescence microscope. Normal nuclear structure in control cells was displayed as green fluorescence, whereas it was bright green in early apoptotic cells caused by interposition of acridine orange with the fragmented DNA. After 24 h, nuclear chromatin pucker and membrane zeiosis were detected as moderate apoptotic features. After 48 h, the reddish-orange color due to binding of propidium iodide to denatured DNA identified the late stage of apoptosis (Supplementary Figure 3).

### Evaluation of reactive oxygen species production

To evaluate the ROS production in the WiDr and HT-29 cells treated with NTC for 24 h, DHE dye was used for staining the live cells after NTC treatment. Following a rapid oxidation of DHE and producing DCF by ROS, the fluorescent intensity was identified by Radiance 2100 confocal microscope (Bio-Rad, Hercules, CA, USA). The DCF fluorescence levels in the cells were remarkably increased in a dose-dependent manner (Supplementary Figure 4).

### Cytotoxic potential of NTC on releasing of LDH

The potential of cytotoxic effect of NTC on cancer cell lines was analyzed at different concentrations after 24 h. The NTC significantly induced release of lactate dehydrogenase. This enzyme is a biomarker of the loss of membrane integrity, apoptosis and necrosis. Results revealed occurrence of cytotoxicity at a concentration of 6.0 μM after 24 h (Supplementary Figure 5).

### NTC mediated NF-κB translocation

Substantial suppressive effect against translocation of TNF-α-stimulated NF-κB in WiDr and HT-29 cells was identified at 6.0 μM of NTC (Figure 5). Non-stimulated state was distinguished by the high NF-κB fluorescence intensity in the cytoplasm of normal cells. High fluorescence intensity was also observed in the nucleus of cancer cells. NTC Activates apoptosis by preventing the activation of NF-κB and its subsequent translocation to the nucleus.

**Figure 5:** **Translocation of NF-κB**. After treatment of both cancer cells by several concentration of NTC for duration of 3 h, the cells were exposed for 30 min to TNF- α (1 ng/ml). Results disclosed no significant cytoplasmic to nucleus translocation of NF-κB. All data were expressed as the means ± standard error of triplicate measurements. ^*^P < 0.05 compared with the no-treatment group.

### NTC upregulated expression of gluthatione reductase

To identify the expression of the genes involved in cellular stress response in the WiDr and HT-29 cells treated with NTC, real time profiler qPCR-array was used. In this method, 84 human genes involved in the oxidative stress and antioxidant defense, antioxidant peroxiredoxin (PRDX) family and redox control were examined. Results showed that the oxidative stress and antioxidant-related genes were differentially expressed in the cells in response to NTC. Interestingly, glutathione reductase was significantly up-regulated >80-fold in both cancer cells as compared with normal cells (*P* < 0.05). This finding was confirmed with further independent qPCR (Supplementary Figure 6).

### NTC induced caspase-3/7, -8, and, -9

The bioluminescent intensity of caspase-3/7, 8 and 9 activities of NTC treated cells were measured at 6, 12, 18, 24, 30, 36, and 42 h time points. Significant increases in caspase-3/7, 8, and 9 activities was detected in the colon cancer cells after 18 and 24 h of NTC exposure (Figure 6). The highest activity for caspase-9 was observed in both cancer cell lines after 18 h of treatment with NTC (5-folds for both cancer cells). After 24 h of NTC exposure caspase-3/7 and 8 activities were increased to a peak in both cancer cell lines and then gradually decreased at the later time points, suggesting that NTC induces apoptosis in WiDr and HT-29 through activation of caspase-9 and 8. Vis-a-vis, addition of caspase inhibitor, Z-VAD-FMK (10 μM) inhibited caspase 3/7, 8, and 9 activities in the presence of 6.0 μM NTC.

**Figure 6:** **Time-dependent activation of caspase 3/7, 8 and 9 by NTC (6.0 μM)**. The results disclosed a significant activation in caspase 3/7, 8, and 9 in a time-dependent manner. All data were expressed as the means ± standard error of triplicate measurements.

### NTC induced both mitochondrial and extrinsic pathways

Western blot analysis revealed a dose-dependent reduction of Bcl-2 (26 KDa) and Bcl-xL (30 KDa) expression levels in WiDr and HT-29 cells treated with NTC. In both colon cancer cell lines, the levels of Bcl-2 and Bcl-xL proteins were substantially altered at 6.0 μM NTC (Figure 7). In addition, upregulation of p53 (53 KDa) and Bax (23 KDa), cleavage of Bid (22 KDa) to its truncation (15 kDa) as well as cleavage of caspase-7 (20 KDa), 8(43 KDa), and 9(37 KDa) were evident in both cell lines. Caspase 3 (17 and 11 kDa subunits) cleavage was detected in cancer cells treated with NTC, but was not seen in normal cells with the similar treatment dosages (Figure 7). This finding suggests that NTC induces apoptosis through both mitochondrial and extrinsic pathways. The NTC also modulates binding of truncated Bid to Bax resulting in the release of cytochrome c from mitochondria.

**Figure 7:** **Western blot analysis of cancer and normal cell lines**. Cells were treated with 3.0 and 6.0 μM of NTC for 24 h. Proteins were transferred to a membrane and followed by probing with antibodies. Normalization of band densities of treated samples were accomplished based on the control. The results represent significant increase in the expression level of caspase 3, 7, 8, 9, p53, Bax and conversion of Bid to its truncated, whereas decrease in Bcl-2 and Bcl-xL level.

### Detection of apoptosis

Cells were pre-treated with cell membrane permeable calcium chelator EGTA/AM (25 μM) for 1 h followed by addition of NTC (6.0 μM) for 24 h. Cells were stained with Annexin V FITC and PI then subjected to flow cytometry analysis. Our data indicates that apoptosis induction by NTC occurred even in the presence of the calcium chelator (Figure 8). This finding suggests that NTC initiates caspase 8 activation and apoptosis independent from calcium signaling.

**Figure 8:** **Quality assay of apoptosis**. Cells were treated with EGTA/AM (25 μM) prior to exposure to NTC 6.0 μM. Apoptosis analysis shows (Left to right); the untreated cells as the control; 24 h NTC-treatment of the cells; 24 h NTC-treatment+ EGTA/AM.

## Discussion

Initiation and progression of cancer is mostly coupled to defective or inefficient apoptosis in normal cells. Therefore, discovery of target selective therapeutic drugs is associated to the comprehensive conception of apoptotic signaling pathways. The cytotoxic properties of nickel(II) complex against colon cancer cell lines were evaluated throughout the current study. Particularly, the NTC was able to initiate a simultaneous activity of mitochondrial and extrinsic pathways of apoptosis in colon cancer cells. The NTC selectively displayed a potent suppressive effect against cancer cells with insignificant influence on normal cells. This phenomenon is affirmed as a significant feature of nickel complexes in the treatment of cancer. To sum up, the cytotoxic effect of NTC against colon cancer cells is associated with both extrinsic and intrinsic apoptotic-dependent signaling pathways. Morphological and biochemical alterations are the two significant events of apoptosis. Following inducing signals in the cell, morphological modifications such as cell shrinkage, chromatin condensation, membrane blebbing, and nuclear fragmentation appear which subsequently form apoptotic bodies. In this study, analysis of the cell membrane permeability, LDH and cytochrome C release, cytoskeleton rearrangement, generation of ROS, mitochondrial membrane potential, nuclear fragmentation and NF-κB translocation was carried out to investigate the NTC-induced cytological changes in colon cancer cells. Results showed that NTC can stimulate cytoskeleton shrinkage-related reorganization. In addition, the NTC, at a concentration of 6.0 μM, substantially damaged membrane integrity and subsequent releasing of LDH from the cells (Supplementary Figure 5). Morphological alterations relevant to the apoptosis was examined through analysis of membrane blebbing and chromatin condensation by using AO/PI staining (Supplementary Figure 3; Aarts et al., 2012). By increasing the period of the cell exposure to NTC from 24 to 72 h, modifications of the early to the late stage of apoptotic events appeared (Gasparri et al., 2006; Tentner et al., 2012; Wang et al., 2012). Cell cycle distribution was verified by using BrdU and phospho-histone H3 staining (Gasparri et al., 2006; Tentner et al., 2012; Wang et al., 2012). Results showed that neither BrdU attachment nor H3 staining in the mitotic stage indicates any remarkable changes of the cell number in S/M phase. Subsequent flow cytometry examination showed that cell arrest occurred at the G1 phase. This finding confirms that cell death was triggered by apoptosis (See et al., 2010; Liu et al., 2012). Mitochondria controls the fate of the cells via shifting in the level of ROS. Based on our data, an elevated level of ROS in the NTC-treated cells (6.0 μM) was determined. This process is controlled through upregulation of GR as shown by qRT-PCR. GR is an oxidative stress indicator and plays a significant role in the scavenging of reactive oxygen species and anti-oxidant function. Enhanced ROS production by NTC could stimulate de novo synthesis of GR (Wu et al., 2004). Disproportionate ROS production diminishes mitochondrial membrane potential leading to the release of cytochrome c from mitochondria into the cytoplasm. Increased mitochondrial cytochrome c levels in the cytoplasm is a key initiative signal for induction of intrinsic apoptosis pathway at 6.0 μM NTC (Bishayee et al., 2013; Zhang et al., 2013). Thus, NTC can be said to be a potential inducer of morphological modifications downstream of apoptotic molecular events in the colon cancer cells associated with its cytotoxic potential.

The apoptosis mechanism is specified by a series of morphological modifications which are triggered by various molecular events to undergo cell death rather than its recovery. Previous studies have demonstrated the cytotoxic effect of some nickel containing compounds such as nickel complex of thiosemicarbazones, nickel(II) complexes with furanylmethyl and thienylmethyl dithiolenes [1,3-dithiole-2-one and 1,3-dithiole-2-thione], nickel chelates of 5-dimethylaminomethyl-2-thiouracil (Afrasiabi et al., 2005; Chohan et al., 2006). To further support the role of NTC in cell death scenarios, we analyzed the apoptotic pathways in the colon cancer cell lines. Results showed that NTC enhanced the release of mitochondrial cytochrome c which activated caspase 9 by 3-folds in colon cancer cells. Interestingly, activated caspase-8 is also increased by 2-folds in cancer cells, suggesting that NTC-induced apoptosis is mediated by more than one pathway. Following cell excitation, calcium ions are released from mitochondria to regulate several cellular processes such as apoptosis. Apoptosis can be directed by calcium signaling. Furthermore, this ion plays an essential role in the control of cell death, although calcium overload is associated with the necrosis. Therefore, prolonged elevation of cytosolic calcium ions causes cell death (Chou et al., 2010). In addition, mitochondrial calcium ion uptake alters the mitochondrial permeability which activates apoptosis events in response to the stress (Gerasimenko et al., 2002). Our data shows that addition of EGTA/AM, diminishes cytosolic calcium ion in both early and late stages of apoptosis within the cancer cell lines (Figure 8). This finding suggests that NTC initiates apoptosis independent from calcium signaling. Calcium chelator (EGTA/AM) application and flow cytometry analysis of Annexin-V in the NTC- treated cells demonstrated the absence of cytosolic free calcium and increased the number of cells. Hence NTC can activate caspase 8 independently from intracellular calcium ion concentrations.

Resistance of colon cancer to chemotherapy is linked to the modification of the interconnection of apoptosis and NF-κB pathways (Park et al., 2015). The process of apoptosis is regulated by NF-κB signaling pathway (Bkarett and Gilmoer, 1999). The B-cell lymphoma 2 (Bcl-2), Bcl extra-large (Bcl-xl), p53, caspase-8, and BH3 interacting-domain death agonist (Bid) are important elements of mitochondria-dependent apoptotic response to drugs. Both Bcl-2 and Bcl-xl belong to the anti-apoptotic Bcl-2 family, the trans-membrane proteins in the mitochondria. Bcl-xl can block cell death through maintenance of mitochondrial homeostasis and Bcl-2, as a checkpoint assists the implementation of caspase cascade (Vander Heiden et al., 1997; Opferman, 2008). Expression of Bcl-2 can be reduced by P53, an apoptosis mediator. Damage of DNA activates p53 to trigger apoptosis and eliminate the permanently injured cells (Ermolaeva and Schumacher, 2014). Defect of Bcl-2, Bcl-xl, and p53 contributes to tumor development and resistance of the cells to chemotherapeutic response (Hassan et al., 2014). Some cytotoxic drugs can also induce caspase-8 to convert Bid to its translocation form (tBid) leading to the release of mitochondrial cytochrome c into the cytoplasm and then activating Bax (Gu et al., 2005; Schug et al., 2011). Results of the current study prove that NTC potentially reduces the levels of Bcl-2 and Bcl-xl, but increases p53 concentration in the colon cancer cells. Moreover, NTC induces the process of cell death through upregulation of Bax and caspase-8/Bid pathway in the colon cancer cell lines. In contrast, the NTC did not activate the NF-κB pathway. This finding supports previously reported data showing that enhanced activity of NF-κB pathway contributes to resistance to anticancer drugs (Bishayee et al., 2013; Shakibaei et al., 2013). NF-κB antagonists could inhibit binding of this molecule to DNA resulting in suppression of cell proliferation. Together, NTC exerts cell death potential through inducing apoptotic pathways and declining the NF-κB pathway.

## Conclusion

Evaluating the cytotoxic properties of NTC in the current study suggests that this compound has potential apoptosis induction ability against colon cancer cells. NTC simultaneously induces both internal and external apoptosis pathways, and hence, can be nominated as a potential anti-cancer agent for future *in vivo* studies.

## Author contributions

The authors whose names are listed immediately below report the following details of affiliation or involvement in an organization or entity with a financial or non-financial interest in the subject matter or materials discussed in this manuscript: NS, NM, MK, SM, AM, NA, GA, BH.

### Conflict of interest statement

The authors declare that the research was conducted in the absence of any commercial or financial relationships that could be construed as a potential conflict of interest.

## Supplementary material

Supplementary Figure 1 **Cytoskeletal rearrangement potential of NTC**. Cells were treated with various concentration of NTC for 24 h with following fixation and staining with Hoechst 33342 and phalloidin. Dose dependent increase of phalloidin intensity was observed in both WiDr and HT-29 cells. Bar charts are showing the average fluorescence intensity of phalloidin. All data were expressed as the means ± standard error of triplicate measurements. ^*^*P* < 0.05 compared with the no-treatment group.

Supplementary Figure 2 **Nuclear DNA fragmentation occurs by NTC treatment**. Cells were treated with NTC (6.0 μM μ/ml) for 24 h which followed by fixation and staining using Hoechst 33342. DNA fragmentation is indicated by red circles.

Supplementary Figure 3 **AO/PI double-staining**. Figure reveals that untreated cells remained healthy after 72 h. Moreover, early apoptotic features such as chromatin condensation and blebbing were witnessed after 24 and 48 h. However, after 72 h of NTC treatment (6.0 μM), late apoptosis event was observed. A, Blebbing of cell membrane; B, Late apoptosis; C, Chromatin condensation; D, Viable cells.

Supplementary Figure 4 **Production of ROS based on the effect of NTC (6.0 μM)**. Formation of ROS was significantly increased in both cancer cell lines. All data were expressed as the means ± standard error of triplicate measurements. ^*^*P* < 0.05 compared with the no-treatment group.

Supplementary Figure 5 **Cytotoxic evaluation of NTC using lactate dehydrogenase (LDH) assay**. Bar charts represent that NTC was significantly able to elevate the release of LDH at the concentration of (6.0 μM). All data were expressed as the means ± standard error of triplicate measurements. ^*^*P* < 0.05 compared with the no-treatment group.

Supplementary Figure 6 **Results showed that glutathione reductase was significantly up-regulated >80-fold in both cancer cells as compared with normal cells (***P*** < 0.05)**.
